The article "On the correlation among the students’ epistemic cognition, academic emotions, and academic achievement in higher education" was retracted in 2025. Reasons: plagiarized text; unreliable results or conclusions; concerns about the citations.

# On the correlation among the students’ epistemic cognition, academic emotions, and academic achievement in higher education

**DOI:** 10.1016/j.heliyon.2024.e30770

**Published:** 2024-05-06

**Authors:** Xiangyang Li, Zhiyong Liu, Linchong Ji

**Affiliations:** College of Art and Design, Yangzhou University, Yangzhou, 225009, China

**Keywords:** Academic emotions, Epistemic cognition, Academic achievement, Chinese undergraduate students, Higher education

## Abstract

Students' academic achievement relies on a variety of pedagogical, affective, and individual factors. The investigation of academic emotions and epistemic cognition has been a focal point in existing research. Previous studies have predominantly delved into the essence of students' epistemic cognition and academic emotions. Nonetheless, the correlation between the epistemic cognition, academic emotions, and academic success of Chinese undergraduate students remains inadequately explored. This research delves into the interconnectedness of these variables and examines which facets of epistemic cognition and academic emotions can forecast students' academic performance. A total of three hundred and eighty (380) Chinese undergraduate students were chosen via random sampling for this study. Their self-reported academic achievements were taken into account. Additionally, they completed questionnaires tailored to evaluate their epistemic cognition and academic emotions. The participants' scores underwent Pearson correlation and multiple regression analyses. The findings indicate that positive emotions correlate positively, while negative emotions correlate negatively with students' academic success. Furthermore, positive emotions and three categories of epistemic cognition were found to be predictors of students' academic accomplishments. In conclusion, it is deduced that both epistemic cognition and positive emotions play a role in enhancing students' academic success. The implications of these findings extend to educational psychologists, educators, and students, both theoretically and practically.

## 1 Introduction

Higher education plays a pivotal role in shaping students as prospective human resources capable of addressing societal challenges [1,2]. Acting as a catalyst for change, higher education not only enhances livelihoods but also fosters social stability [1]. At the micro-level, higher education is closely linked to improved living standards by boosting productivity. Research suggests that individuals who attain a quality higher education experience greater social and economic prospects [[1], [2], [3], [4]]. Education serves as a conduit for nurturing skilled and knowledgeable human capital, often regarded as the driving force behind economic growth, consequently propelling the development of nations [3]. Nonetheless, the acquisition of knowledge, values, skills, and attitudes through education is a laborious and intricate process [1,2]. Achieving the goals and missions of higher education demands considerable time and effort from students, with academic achievement influenced by various factors [5].

The article "On the correlation among the students’ epistemic cognition, academic emotions, and academic achievement in higher education" was retracted in 2025. Reasons: plagiarized text; unreliable results or conclusions; concerns about the citations.

Academic accomplishment pertains to the extent to which a learner achieves their educational goals, whether immediate or long-range, commonly assessed by means of metrics like cumulative grade point average (CGPA) or continuous evaluations [6]. Students who attain high levels of academic achievement often enjoy increased income, improved employment perks, and greater prospects for career advancement [6]. Furthermore, individuals with a track record of academic success tend to exhibit heightened levels of self-assurance and self-worth, alongside reduced levels of depression and anxiety [7].

As a critical determinant of university students' access to social and economic opportunities, students' academic achievement depends on many cognitive, affective, and educational variables. Hence, it is imperative to identify the primary factors that contribute to and are associated with academic success [8]. Various elements influence the academic performance of students within educational settings [9], encompassing academic emotions linked to motivational, cognitive, physiological, and behavioral mechanisms [10,11]. The control value proposed by Pekruns [11] offers scholars a robust framework for investigating the effects of various emotions that students encounter within educational settings. This theoretical perspective posits that students' emotions and academic achievement are influenced by expectancy-value theories, attributional theories, and performance models. This theory assumes that expectancy-value theories of transactional approaches, attributional theories, and performance models affect the students' emotions and achievement. It is also assumed that different emotions, particularly academic emotions, are associated with the students' academic outcomes [4]. Yu and Dong [13] have maintained that the student's academic emotions affect their academic achievements manifested while doing the daily homework, learning in classrooms, and taking exams. Researchers have classified academic emotions in different ways. Nevertheless, the predominant typology employed to classify academic emotions indicates that positive and negative emotions can be categorized as either activating or deactivating: Positive/Negative Activating Emotions (PNAE) and Positive/Negative Deactivating Emotions (NADE) [10]. This framework has been commonly utilized by academics and researchers with a focus on academic emotions [[11], [12], [13], [14], [15], [16], [17]].

The article "On the correlation among the students’ epistemic cognition, academic emotions, and academic achievement in higher education" was retracted in 2025. Reasons: plagiarized text; unreliable results or conclusions; concerns about the citations.

Prior research has primarily overlooked the interplay between academic achievement and academic emotions [9]. Strikingly, certain scholars have argued that positive emotions could potentially impede students' academic success, while negative emotions might paradoxically bolster academic achievement [18]. Wang and Chen [19] propose that this phenomenon may arise from positive high-arousal emotions boosting students' complacency, whereas negative emotions could transform pressures into motivational drivers for learning. Despite the pivotal role of emotions in academic environments, scant attention has been directed towards examining the link between students' positive and negative emotions and their academic performance. Hence, there is a pressing need to explore the correlation between students' academic emotions and academic achievement, particularly among a substantial cohort of undergraduate students in China.

Another variable that might contribute to the student's academic achievement is their epistemic cognition, introduced by Hofer [20]. Epistemic cognition is about both theories and beliefs. It is also about how the students define, acquire, and use knowledge [e.g., 21, 22,23]. Within this concept, epistemic cognition deal with knowledge and knowing, constituting coherent epistemic theories [14] as an integral part of epistemic cognition. Researchers interested in developmental psychologists have studied the association between individuals' epistemological beliefs and their educational progress [5]. Similarly, educational psychologists have studied how students' beliefs in knowledge affect the students' learning and academic achievement [5,12,13].

This study delves into the critical role of higher education in shaping students as future contributors to community problem-solving, emphasizing its potential as a catalyst for positive change, improved livelihoods, and enhanced social stability. Acknowledging the intricate nature of the educational journey, the study posits that academic achievement, measured through cumulative grade point averages (CGPA) or continuous assessment, serves as a pivotal factor in determining students' access to social and economic opportunities. Notably, good academic performance is linked to higher incomes, better employment benefits, increased self-confidence, and lower levels of depression and anxiety. To comprehend the multifaceted factors influencing academic achievement, the study explores the relatively unexplored relationship between academic emotions (both positive and negative) and student performance, employing a typology that distinguishes between activating and deactivating emotions. Additionally, the investigation delves into the impact of students' epistemic cognition, encompassing theories and beliefs about knowledge, on academic achievement. By addressing these gaps in previous research, the study aims to provide valuable insights for educational psychologists, faculty, and students. This study investigates whether and which academic emotions are associated with university students' academic achievement. This study also focuses on the association between the students' epistemic cognition and academic achievement.

The article "On the correlation among the students’ epistemic cognition, academic emotions, and academic achievement in higher education" was retracted in 2025. Reasons: plagiarized text; unreliable results or conclusions; concerns about the citations.

### 1.1 Research objectives

The examination of the pertinent literature indicates a plethora of studies that concentrate on the academic emotions, epistemic cognition, and academic accomplishments of university students. Nevertheless, there exists a necessity for a more intricate analysis of the correlation among the academic emotions, epistemic cognition, and academic achievements of university students. The primary aim of this research is to further explore this correlation by examining the link between students' academic emotions and their academic achievements. Moreover, it seeks to explore the connection between students' epistemic cognition, its various elements, and academic achievements. To direct this exploration, the study addresses the following research inquiries.

1. Is there any statistically significant correlation between university students' academic achievement and their academic emotions?
2. Which component of academic emotions more significantly predicts university students' academic achievement?
3. Is there any statistically significant correlation between university students' academic achievement and their epistemic cognition?
4. Which component of epistemological beliefs more significantly predicts university students' academic achievement?

### 1.2 Review of the literature

#### 1.2.1 Academic emotions and academic achievement

Lei and Cui [16] provided a definition of academic emotions as the emotional experiences of students in relation to the educational processes of teaching and learning, encompassing emotions like enjoyment, hopelessness, boredom, anxiety, anger, and pride (p.1541). Academic emotions have been categorized into four groups based on arousal and enjoyment principles: positive low-arousal, negative low-arousal, and negative high-arousal [17]. The argument is also made that achievement emotions consist of both prospective emotions, such as fear of failure, and retrospective emotions, for instance, shame, which students encounter following the receipt of feedback on their academic accomplishments.

The article "On the correlation among the students’ epistemic cognition, academic emotions, and academic achievement in higher education" was retracted in 2025. Reasons: plagiarized text; unreliable results or conclusions; concerns about the citations.

Academic achievement is a frequently used criterion for evaluating education systems, teachers' effectiveness, schools, and student failure or success changes [1,2]. Therefore, researchers interested in the field investigated the causal relationship between the students' academic emotions and academic attainment through a body of practical studies [24,25]; however, inconsistent results have been found. In general, it is expected that positive emotions predict positive consequences in academic contexts, like high grades and good performance on local and large-scale educational evaluations [26,27]. However, we expect negative emotions to be associated with negative consequences such as low grades and impaired performance in the classroom and standard examinations [28,29]. Positive emotions (hope, enjoyment, and pride) serve to enhance the student's curiosity and determination towards the learning process, fostering active participation, stimulating the adoption of innovative learning approaches, and facilitating the demonstration of self-regulated learning. Conversely, negative emotions like hopelessness, shame, anxiety, and boredom detrimentally impact students' motivation, enthusiasm, interest, and dedication to learning, leading to the utilization of rote learning methods instead of profound and significant learning practices that necessitate students' full engagement in the educational journey [11].

The Chinese version of the Academic Emotions Questionnaire was developed by Dong and Yu [12] with a specific focus on assessing academic emotions in adolescents. Academic emotions have been associated with various elements such as cognitive engagement, learning incentives, and methodologies. Lei and Cui's meta-analysis findings [15] offered support for the positive connections between positive high-arousal, positive low-arousal, and academic performance, as well as the negative correlations between negative high-arousal, negative low-arousal, and academic achievement. The scholars suggested that variables like student age, geographical location, and gender may act as moderators in the influence of epistemic cognition on academic achievement.

#### 1.2.2 Students’ epistemic cognition

Epistemology is a psychological concept associated with the fundamental aspects of knowledge, reasoning, and conceptions regarding knowledge's nature and core [30]. The focus in epistemic cognition is on the process through which students acquire knowledge, contemplate knowledge, and shape their understanding of their surroundings [31,32]. Within academic literature, Shirzad et al. [33] have introduced various terms such as epistemic cognition, epistemological reflection, reflective judgment, epistemological resources, and personal epistemologies to denote the concept of epistemic cognition. Schommer [33] has proposed diverse perspectives on the origin of knowledge, highlighting three distinct dimensions: the certainty of knowledge, knowledge as an absolute entity, and the speed of knowledge acquisition.

The article "On the correlation among the students’ epistemic cognition, academic emotions, and academic achievement in higher education" was retracted in 2025. Reasons: plagiarized text; unreliable results or conclusions; concerns about the citations.

Reviewing the existing studies on epistemic cognition reveals different phases [[34], [35], [36], [37], [38]]. The initial phase of studies commenced with qualitative inquiries, primarily examining the concept of epistemic cognition [20]. Notably, Perry [39] outlined the epistemological evolution of college students, noting a progression from perceiving knowledge as absolute truths to embracing relativistic perspectives, and eventually to acknowledging knowledge as an amalgamation of interpreted viewpoints [20] (p.777). Epistemic cognition is commonly classified into three primary categories: relativism, absolutism or dualism, and evaluations or integrated thinking [23].

The subsequent phase of research on epistemic cognition aimed to quantify this phenomenon through Likert scales, predominantly employing mixed methods research [40]. For instance, Lonka et al. [51] investigated the correlation between epistemic cognition and comprehension standards among medical and psychological students. Their findings indicated a connection between epistemic cognition and students' learning approaches. Similarly, Tsai and Liu [42] synthesized studies on science education, concluding that students who perceive scientific knowledge as constructed by scientists (a relativistic standpoint) are more inclined to adopt effective science learning strategies.

Moreover, epistemic cognition has been identified as a significant factor influencing students' goal-oriented performance, despite variations in students' epistemic cognition and the learning strategies they utilize [43,44]. A similar observation was made by Arslanta [45], suggesting a reciprocal relationship between students' epistemic cognition and their learning strategies. Furthermore, a meta-analysis of 132 non-experimental studies conducted by Greene et al. [46] demonstrated a positive correlation between epistemic cognition and academic success (r = 0.162, p < 0.001), albeit the correlation coefficient being modest, the association was statistically significant.

Researchers [36,37,39] have argued that disparities in students' epistemic cognition impact various educational outcomes for both students and educators, particularly influencing students' academic performance [46], self-regulated learning [47], and grasp of scientific concepts [48], alongside numerous other educational characteristics and variables.

The article "On the correlation among the students’ epistemic cognition, academic emotions, and academic achievement in higher education" was retracted in 2025. Reasons: plagiarized text; unreliable results or conclusions; concerns about the citations.

Lin et al. [49] have reported that students with complex epistemological beliefs use mixed motivation and learning strategies. However, learners who believe in the certainty of knowledge use surface learning strategies and have surface motivation. Recently, Guo et al. [50] examined the relationship between reflective thinking and epistemological beliefs. They concluded that epistemological beliefs affect the students’ interest and reflective thinking.

## 2 Materials and methods

### 2.1 Participants

Approximately 420 senior undergraduate students from various faculties within Yangzhou University (YZU) were initially enlisted, yet only 380 students completed and returned the distributed questionnaires. Consequently, the final sample size for this investigation was established at 380. Examination of participants' self-disclosures indicated an age range spanning from 20 to 30 years (M = 25.36, SD = 2). Permission for participation was obtained from both the students and university authorities, with all students opting to voluntarily engage in the survey. The cohort comprised individuals drawn from senior undergraduate cohorts across disciplines such as humanities and social sciences (n = 90), natural sciences (n = 80), engineering (n = 70), agriculture (n = 80), and medicine (n = 60), all of whom were Chinese native speakers. Gender distribution among participants revealed 180 females and 200 males. All participants were duly informed about the study's objectives and duly completed informed consent documentation. They were assured of the confidentiality of collected data and that their responses would bear no consequence on their academic standing within the university.

### 2.2 Measures

In this investigation, three tools were utilized to comprehensively evaluate critical elements of students' educational encounters. The primary tool employed was a self-administered questionnaire crafted to collect information on students' academic accomplishments, with a specific focus on their overall Grade Point Average (GPA). Participants were presented with a variety of grading classifications, ranging from A (90–100 %) to F (Failure, 0–59 %), along with corresponding percentage intervals. After completion, the documented grades were transformed into numerical values for subsequent examination.

Epistemic cognition, an essential aspect of students' cognitive processes, was assessed utilizing the Epistemic Cognition Scale. This scale, comprising 15 Likert-type statements, was adapted from the MED NORD questionnaire, which was initially formulated and authenticated by Lonka et al. (2008). It gauged different facets of epistemic cognition, such as reflective learning, collaborative knowledge construction, appreciation of metacognition, certainty in knowledge, and practical utility. Participants assigned a rating to each statement on a six-point Likert scale, offering insights into their cognitive strategies for learning. The scale's internal consistency was evaluated through Cronbach's alpha coefficient, demonstrating values between 0.81 and 0.88, indicating dependable reliability across its elements.

The article "On the correlation among the students’ epistemic cognition, academic emotions, and academic achievement in higher education" was retracted in 2025. Reasons: plagiarized text; unreliable results or conclusions; concerns about the citations.

Additionally, the academic emotions of participants were scrutinized through the Academic Emotion Questionnaire (AEQ), devised and authenticated by Pekrun et al. (2005). This questionnaire consisted of 75 statements aimed at capturing eight specific emotions encountered by students in academic environments. These emotions spanned from positive (pride, hope, joy) to negative (anger, boredom, shame, fear, hopelessness) and were assessed on a 5-point Likert scale. Cronbach's alpha coefficients were calculated to assess the internal consistency of each emotional dimension, yielding values between 0.78 and 0.89, indicating reliable consistency across the emotional spectrum.

### 2.3 Procedure

A correlational research method was employed to answer the research questions. First, admission to enter the university and the classrooms was obtained from the university administrators and teachers. The students were recruited and asked to fill in the informed consent forms. Then, they were required to fill in the questionnaires and the self-report scale for cumulative GPA. That is, each participant reported the cumulative GPA for all courses passed during the last semesters. Each participant was coded numerically, and the questionnaires without missing data were coded and entered into SPSS. Data were analyzed in different ways. The mean scores and standard deviation for each variable were estimated. The assumptions of multiple regression analysis including Linearity, Homoscedasticity, lack of outliers, normality of residuals, and independence of residuals were all checked and none of them was violated. In addition, the correlation coefficient between the variables was estimated (p = 0.05). Finally, two multiple regression analyses were run.

### 2.4 Ethical considerations

This study received ethical approval from the Ethics Committee of Yangzhou University (Number: YU 23465). The research protocol was carefully reviewed to ensure compliance with all relevant regulations and standards of ethical considerations. Approval was granted after confirming that the study posed no adverse effects on the participants. Prior to their involvement, all participants were provided with informed consent forms, which they were required to read, understand, and sign. They were assured that participation was voluntary and that they had the right to withdraw from the study at any stage without any consequences.

The article "On the correlation among the students’ epistemic cognition, academic emotions, and academic achievement in higher education" was retracted in 2025. Reasons: plagiarized text; unreliable results or conclusions; concerns about the citations.

## 3 Results

Four hundred twenty senior undergraduate students completed the questionnaires (self-report academic achievement, academic emotions, and epistemic cognitions). Forty questionnaires were excluded from the final analysis due to missing data, and participants were required to respond to all items. Ultimately, 380 questionnaires were deemed valid (180 females and 200 males). The age of the students ranged from 20 to 30 years. The data analysis commenced with the computation of mean scores and standard deviation (SD), conducting Pearson correlations among the variables and correlation matrix for all measured variables, as well as multiple regression analysis. The findings, encompassing both descriptive and inferential statistics, are presented in a sequential manner.

### 3.1 The students’ academic emotions and academic achievement

The relationship between academic achievement and academic emotions in undergraduate students was examined in this study. The findings (Table 1) demonstrated a statistically significant (p < 0.01) correlation between academic achievement (GPA) and enjoyment (r = 0.37), hop (r = 0.27), pride (r = 0.39), and hop. On the other hand, there was a negative (p < 0.01) correlation between academic achievement and negative emotions such as shame (r = −0.21), boredom (r = −0.21), anxiety (r = −0.24), hopelessness (r = −0.23), and anger (r = −0.15). Results are shown in Table 1.

**Table 1:** Correlation Matrix of academic emotions and academic achievement.

	1	2	3	4	5	6	7	8	9	M/SD
1. Enjoyment	1									3.7/0.7
2. Hope	0.38	1								3.6/0.61
3. Pride	0.46	0.77	1							4.1/.81
4. Anger	−0.07	−0.06	0.09	1						2.9/0.61
5. Anxiety	−0.27	−0.10	0.13	0.39	1					2.1/0.63
6. Hopeless	−0.09	0.10	--0.06	0.45	0.77	1				2.3/0.61
7. Shame	−0.19	−0.09	−0.10	0.39	0.87	0.79	1			2.4/0.54
8. Boredom	−0.14	−0.30	−0.29	−0.43	0.81	0.91	0.67	1		2.5/0.6
9. GPA	0.37	0.27	0.39	−0.15	−0.24	−0.23	−0.215	−0.21	1	75/11

Note. p < 0.05.

The scores of the participants on positive and negative emotions were analyzed using multiple regression analysis to investigate the anticipatory impact of each independent variable (academic emotions and motivation) on the dependent variable (academic performance of students). Findings revealed that positive emotions (β = 0.117) were notably influential in predicting academic performance, explaining 40 % of the variability in academic performance (refer to Table 2).

The article "On the correlation among the students’ epistemic cognition, academic emotions, and academic achievement in higher education" was retracted in 2025. Reasons: plagiarized text; unreliable results or conclusions; concerns about the citations.

**Table 2:** Multiple regression for predicting academic achievement based on academic emotions and motivation.

Model	Unstandardized coefficients	Standardized coefficients		F	R	R^2^	T	P
	B	SE						
Constant	11.98	0.88					14.11	0.001
Positive emotions	0.467	0.240	0.118	49.56	0.64	0.41	1.98	0.041
Negative emotions	−0.081	0.13	−0.031				0.62	0.581

The multiple regression analysis was conducted to assess the predictive value of academic emotions and motivation on academic achievement. The findings revealed that positive emotions significantly contributed to academic achievement (B = 0.467, β = 0.118, t = 1.98, p = 0.041). The positive unstandardized coefficient indicates that, on average, for each one-unit increase in positive emotions, academic achievement is expected to increase by 0.467 units. The standardized coefficient (β) of 0.118 suggests a positive relationship between positive emotions and academic achievement, even after controlling for other variables. This effect was statistically significant at the 0.05 level. Conversely, negative emotions did not demonstrate a significant impact on academic achievement (B = −0.081, β = −0.031, t = 0.62, p = 0.581). The unstandardized coefficient of −0.081 implies that, on average, for each one-unit increase in negative emotions, academic achievement is expected to decrease by 0.081 units. However, the lack of statistical significance (p > 0.05) suggests that the relationship between negative emotions and academic achievement is not reliably different from zero.

## 4 Students’ epistemic cognition and academic achievement

The second goal of this study was to measure the correlation between undergraduate students’ epistemic cognition and academic achievement. Correlation results revealed that the components of the epistemic cognition were significantly correlated with academic achievement (p < 0.01). Results are shown in Table 3.

**Table 3:** Correlation Matrix of the epistemic cognition and academic achievement.

	1	2	3	4	5	6	7	M/SD
1. Collaborative knowledge-building	1							3.2/0.61
2. Valuing metacognition	0.46	1						3.1/0.53
3. Practical value	0.55	0.49	1					3.2/0.62
4. Reflective learning	0.32	0.23	0.32	1				3.4/0.58
5. Certain knowledge	0.38	0.32	0.44	0.40	1			3.63/0.71
6. Epistemic cognition (total)	0.88	0.87	0.90	0.87	0.86	1		3.31/0.72
6. GPA	0.24	0.23	0.15	0.38	0.22	0.21	1	75/11

Note. *p < 0.05.

The correlation analysis revealed a significant relationship between GPA and students' epistemic cognition (r = 0.24, p < 0.05). Furthermore, significant correlations were observed between students' academic achievement and various components of epistemic cognition: collaborative knowledge-building (r = 0.24, p < 0.05), valuing metacognition (r = 0.23, p < 0.05), practical value (r = 0.15, p < 0.05), reflective learning (r = 0.38, p < 0.05), certain knowledge (r = 0.22, p < 0.05), and epistemic cognition collectively (r = 0.21, p < 0.01). Upon detailed analysis, it was found that the correlation between reflective learning and GPA (r = 0.38) was stronger compared to the correlation between GPA and other components of epistemic cognition. To further explore the predictive value of different components of epistemic cognition on students' academic achievement, multiple regression analyses were conducted. Results of these analyses are presented in Table 4.

The article "On the correlation among the students’ epistemic cognition, academic emotions, and academic achievement in higher education" was retracted in 2025. Reasons: plagiarized text; unreliable results or conclusions; concerns about the citations.

**Table 4:** Multiple regression for predicting the students’ academic achievement based on epistemic cognition.

Model	Unstandardized coefficients	Standardized coefficients		F	R	R^2^	T	P
	B	SE	B					
Constant	14.98	0.78					16.11	0.001
1. Collaborative knowledge-building	0.56	0.31	0.15	55.61	0.40	0.16	1.98	0.05
2. Valuing metacognition	0.36	0.12	0.10				1.94	0.05
3. Practical value	0.14	0.19	0.09				0.54	0.62
4. Reflective learning	0.43	0.37	0.17				2.3	0.01
5. Certain knowledge	0.091	0.12	0.049				0.71	0.42

The multiple regression analysis aimed to predict students' academic achievement by assessing the impact of various dimensions of epistemic cognition. The results are summarized in the table. The constant term (14.98) represents the baseline academic achievement when all predictor variables are zero. Collaborative knowledge-building beliefs demonstrated a significant positive association with academic achievement (B = 0.56, β = 0.15, t = 1.98, p = 0.05), indicating that, on average, for each one-unit increase in collaborative knowledge-building beliefs, academic achievement is expected to increase by 0.56 units. Similarly, valuing metacognition beliefs were positively associated with academic achievement (B = 0.36, β = 0.10, t = 1.94, p = 0.05). However, practical value beliefs did not yield a statistically significant effect (B = 0.14, t = 0.54, p = 0.62). Reflective learning beliefs exhibited a significant positive association with academic achievement (B = 0.43, β = 0.17, t = 2.3, p = 0.01), suggesting that an increase in reflective learning beliefs is associated with a corresponding increase in academic achievement. Conversely, certain knowledge beliefs did not show a significant association with academic achievement (B = 0.091, t = 0.71, p = 0.42).

## 5 Discussion

The results showed significant positive relationships between students' positive academic emotions, particularly pride, joy, and hope, and their academic performance. Notably, higher levels of pride, joy, and hope were associated with better academic outcomes. This result is consistent with previous research efforts [1,3,4,7,17,[29], [30], [31]]. For instance, a longitudinal study carried out in Germany revealed a similar trajectory and indicated that positive emotions had a predictive function in the “learning performance” of German students [30]. These findings align with control value theory and indicate a significant impact of academic emotions on the academic endeavors of students. The effects are underpinned by diverse mediating mechanisms, encompassing students' self-regulation tactics and their drive to acquire knowledge [22]. As posited by Pekrun et al.'s theory [16], academic emotions wield their impact through various intermediary factors, including metacognitive and cognitive learning approaches, intrinsic and extrinsic motivations, as well as self-regulation techniques. Emotions serve to stimulate heightened cognitive engagement like problem-solving and strategic thinking, while also promoting the utilization of cognitive (e.g., elaboration, organization, strategic thinking, critical thinking) and metacognitive strategies (e.g., regulatory strategies, monitoring). Academic emotions can further incentivize students to surmount obstacles encountered in academic settings by putting in diligent effort, thereby potentially boosting their academic performance [15,22,31,32].

The article "On the correlation among the students’ epistemic cognition, academic emotions, and academic achievement in higher education" was retracted in 2025. Reasons: plagiarized text; unreliable results or conclusions; concerns about the citations.

Positive emotions have the capability to enhance the motivation for learning among students by focusing on the learning process, thereby facilitating the application of learning and self-regulation techniques. Consequently, academic emotions play a crucial role in influencing students' academic performance under specific circumstances. Previous research has demonstrated a noteworthy negative relationship between various negative emotions (e.g., hopelessness, fear, shame, anger, boredom) and students' academic accomplishments. This discovery aligns with the findings of several earlier studies [1,3,29]. Negative emotions, such as hopelessness and boredom, have adverse effects on learning and academic success as they can impede information processing, diminish motivation, and divert students' attention from learning tasks. Furthermore, the outcomes corroborate a longitudinal investigation conducted by Pekrun et al. [33] which indicated that negative emotions like anger, hopelessness, fear, shame, and boredom are indicative of students' final grades. Conversely, according to Pekrun [15], negative emotions diminish students' focus, making it more likely for them to employ superficial learning tactics like rote memorization and rehearsal.

The second objective was to explore the association between undergraduate students' epistemic cognition and academic achievement. It was found that all components of epistemic cognition significantly predict the students' academic performance. Results align with the findings of the meta-analysis study undertaken by Greene et al. [46]. Findings are also consistent with Bromme et al., 2009 who suggest that epistemological beliefs greatly influence the learning process and outcomes mainly by affecting the students' understanding of the learning task and the knowledge they are supposed to acquire.

The article "On the correlation among the students’ epistemic cognition, academic emotions, and academic achievement in higher education" was retracted in 2025. Reasons: plagiarized text; unreliable results or conclusions; concerns about the citations.

The findings of the multiple regression analysis in this study align with and are supported by a rich body of literature investigating determinants of academic achievement and the role of epistemic cognition. Numerous studies have explored factors influencing academic performance across diverse educational settings [[1], [2], [3], [4], [5], [6], [7]], emphasizing the multifaceted nature of achievement.

The positive association between collaborative knowledge-building beliefs and academic achievement resonates with research highlighting the significance of students' collaborative efforts and belief systems in fostering academic success [5]. This finding is consistent with the notion that active engagement in collaborative knowledge construction positively contributes to learning outcomes [5,50]. The positive relationship identified between valuing metacognition beliefs and academic achievement aligns with existing literature emphasizing the importance of metacognitive awareness in students' overall academic success [8]. Metacognition, including the ability to monitor and regulate one's cognitive processes, has been linked to enhanced learning outcomes [8,44].

The non-significant correlation between practical value beliefs and academic achievement corresponds with the nuanced nature of the impact of practical value dimensions across different contexts [1,2]. While some studies emphasize the importance of perceived practical value in academic success, others suggest its limited role in predicting achievement [1,2].

Moreover, the significant positive association between reflective learning beliefs and academic achievement is consistent with the idea that students who engage in reflective practices tend to demonstrate higher academic performance [28]. This aligns with the growing body of literature emphasizing the role of reflective learning strategies in academic success [28]. The lack of significant association between certain knowledge beliefs and academic achievement is in line with the notion that not all dimensions of epistemic cognition may equally contribute to academic outcomes [39,41]. This result underscores the need for a nuanced understanding of how specific cognitive dimensions influence academic success.

The article "On the correlation among the students’ epistemic cognition, academic emotions, and academic achievement in higher education" was retracted in 2025. Reasons: plagiarized text; unreliable results or conclusions; concerns about the citations.

To further contextualize these findings, it is essential to consider the broader literature on academic emotions and their impact on achievement [9,10,[13], [14], [15], [16]]. Positive academic emotions, such as those related to achievement, have been linked to higher academic performance [9,10]. Additionally, the interplay between academic emotions and self-regulated learning behaviors has been explored [17]. These emotional and motivational factors can contribute to a comprehensive understanding of the complex dynamics influencing students' academic achievement [10,16,26].

The overarching framework of epistemic cognition, as discussed in the literature [[20], [21], [22], [23], [24], [25], [26], [27], [28], [29], [30], [31], [32], [33], [34], [35]], provides a theoretical foundation for understanding how students' beliefs about knowledge and knowing may influence their academic outcomes. The current study's focus on specific dimensions of epistemic cognition adds granularity to this framework, offering insights into the differential effects of various cognitive dimensions on academic achievement.

Findings also echo the results of the study by some of the previous studies [51], indicating that epistemic cognition are potent factors influencing students' goal-oriented performance. Therefore, it can be argued that the students' epistemic cognition has effect on their learning strategies, contributing to their academic achievement [52,53]. Findings also support the conclusions made by the previous studies, which indicated that changes in the students' epistemic cognition affect their educational outcomes and academic achievement [47,48] by fostering self-regulated learning [46] and scientific understanding [47,50]. Similarly, it can be argued that students' epistemic cognition led to deep learning strategies and motivation for learning, which greatly affect the students' educational outcomes [49]. Furthermore, in line with Guo et al. [50] findings, epistemological beliefs affect the students’ interest and reflective thinking, affecting their academic competence/achievement [54].

## 6 Conclusions

Several conclusions can be drawn in accordance with the study's findings. The first finding indicates a strong correlation between improved academic performance and positive academic emotions like pride, joy, and hope. These feelings motivate students to overcome academic obstacles, promote the application of efficient learning strategies, and enhance cognitive processing—all of which are in line with earlier research. On the other hand, there is a strong negative correlation between academic achievement and negative academic emotions like hopelessness, fear, shame, anger, and boredom. These emotions cause disruptions in information processing, lower motivation, and encourage superficial learning strategies. The study also shows how important epistemic cognition is in predicting academic performance. Students' perceptions of knowledge and knowing affect how they interpret assignments and how much knowledge they learn, which in turn affects how well they do academically. Academic achievement is positively correlated with collaborative knowledge-building beliefs and metacognitive value, highlighting the significance of metacognitive awareness and cooperative efforts in improving learning outcomes. Reflective learning techniques also have a positive impact on academic performance, highlighting the role that reflective practices play in encouraging greater achievement.

The article "On the correlation among the students’ epistemic cognition, academic emotions, and academic achievement in higher education" was retracted in 2025. Reasons: plagiarized text; unreliable results or conclusions; concerns about the citations.

Furthermore, the nuanced nature of practical value beliefs and certain knowledge beliefs is evident, as they do not show significant correlations with academic achievement in this study. This underscores the need for a nuanced understanding of how specific dimensions of epistemic cognition influence academic outcomes, emphasizing the multifaceted nature of factors influencing students' learning outcomes. Overall, these conclusions contribute to a comprehensive understanding of the complex dynamics between academic emotions, epistemic cognition, and academic achievement. They underscore the importance of addressing emotional and cognitive factors in educational settings to foster student success. Additionally, the findings have theoretical and practical implications for the development of effective educational interventions aimed at promoting positive emotional well-being, fostering metacognitive awareness, and enhancing reflective learning practices to ultimately improve academic outcomes.

This study enjoyed different strengths. First, the study addresses an important and current topic focusing on the relationship between academic emotions, epistemic cognition, and academic performance in university students. This is a relevant issue for the academic community and may have significant implications for improving education. Second, the sample included 380 students from various faculties, contributing to the representativeness of the results. This allows for broad generalization of findings within the university context. Third, the study utilized standardized questionnaires to measure both academic emotions and epistemic cognition. This provides a strong methodological foundation for data analysis and result interpretation. Finally, the study's results indicate significant correlations between academic emotions, epistemic cognition, and academic performance. These findings may have practical implications for improving the teaching and learning process.

The article "On the correlation among the students’ epistemic cognition, academic emotions, and academic achievement in higher education" was retracted in 2025. Reasons: plagiarized text; unreliable results or conclusions; concerns about the citations.

## Limitations and suggestions for further studies

In this study, we were unable to examine the potential correlation between academic emotions and epistemic cognition, despite having access to the necessary data. Future researchers could address this gap by employing structural equation modeling to explore the relationships among students' academic emotions, epistemic cognition, and academic achievement, using a representative sample of participants. Additionally, the study did not include a comparison of students from different academic disciplines in relation to the variables under investigation. It is recommended that other researchers investigate how students' majors influence their academic emotions and epistemic cognition. Another limitation was the researchers' inability to recruit participants from a representative sample of universities in China. To overcome this limitation, it is suggested that future studies replicate the research on a larger scale by including undergraduate, graduate, and postgraduate students, in order to examine whether the academic degree of students moderates the associations between their epistemic cognition, academic emotions, and academic achievement.

## Availability of supporting data

The data will be made available by the authors if requested.

## Data availability statement

The data will available upon the request.

## CRediT authorship contribution statement

**Zhiyong Liu:** Writing – review & editing, Writing – original draft, Formal analysis, Data curation, Conceptualization. **Linchong Ji:** Writing – review & editing, Writing – original draft, Methodology, Investigation.

## Declaration of competing interest

The authors declare that they have no known competing financial interests or personal relationships that could have appeared to influence the work reported in this paper.

## References

[1] Tadese M., Yeshaneh A., Mulu G.B. (2022). Determinants of good academic performance among university students in Ethiopia: a cross-sectional study. BMC Med. Educ..

[2] Idris F., Hassan Z., Ya’acob A., Gill S.K., Awal N.A.M. (2012). The role of education in shaping youth's national identity. Procedia Soc Behav Sci.

[3] Sothan S. (2019). The determinants of academic performance: evidence from a Cambodian University. Stud. High Educ..

[4] Talib N., Sansgiry S.S. (2012). Determinants of academic performance of university students. Pakistan. J. Psychol. Res..

The article "On the correlation among the students’ epistemic cognition, academic emotions, and academic achievement in higher education" was retracted in 2025. Reasons: plagiarized text; unreliable results or conclusions; concerns about the citations.

[5] Mardiha S.M., Alibakhshi G. (2020). Teachers' personal epistemological beliefs and their conceptions of teaching and learning: a correlational study. Cogent Education.

[6] Regier J. (2011). Why is academic success important?. Appl Sci Technol Scholarsh.

[7] Yigermal M.E. (2017). Determinant of academic performance of undergraduate students: in the cause of Arba Minch university Chamo Campus. J. Educ. Pract..

[8] Hayat A.A., Salehi A., Kojuri J. (2018). Medical student's academic performance: the role of academic emotions and motivation. J Adv Med Educ Prof.

[9] Yavorsky K. (2017).

[10] Pekrun R., Goetz T., Frenzel A.C., Barchfeld P., Perry R.P. (2011). Measuring emotions in students' learning and performance: the Achievement Emotions Questionnaire (AEQ). Contemp. Educ. Psychol..

[11] Pekrun R., Frenzel A.C., Goetz T., Perry R.P. (2007).

[12] Pekrun R. (2006). The control-value theory of achievement emotions: assumptions, corollaries, and implications for educational research and practice. Educ. Psychol. Rev..

[13] Dong Y., Yu G.L. (2010). Effects of Adolescents' academic emotion on their academic achievements. Journal of Psychological Science.

[14] Chen J.J., Li S.F. (2012). The paths of junior school students ‘achievement attribution and academic emotions forecasting their academic achievement. Chin. J. Clin. Psychol..

[15] Lei H., Cui Y. (2016). Effects of academic emotions on achievement among mainland Chinese students: a meta-analysis. OCIAL BEHAVIOR AND PERSONALITY.

[16] Pekrun R., Lichtenfeld S., Marsh H.W., Murayama K., Goetz T. (2017). Achievement emotions and academic performance: longitudinal models of reciprocal effects. Child Dev..

[17] Artino A.R., Jones K.D. (2012). Exploring the complex relations between achievement emotions and self-regulated learning behaviors in online learning. Internet High Educ..

[18] Turner J.E., Schallert D.L. (2001). Expectancy–value relationships of shame reactions and shame resiliency. J. Educ. Psychol..

[19] Wang A.P., Chen H.S. (2005). A study on the effects of learning anxiety, learning attitude, and motivation on test performance. Psychol. Dev. Educ..

[20] Hofer B.K., Greene J.A., Sandoval W.A., Bråten I. (2016). Handbook of Epistemic Cognition.

[21] Kitchener K.S. (1983). Cognition, metacognition, and epistemic cognition. Hum. Dev..

[22] Kuhn D., Weinstock M., Hofer B.K., Pintrich P.R. (2002). Personal Epistemology: the Psychology of Beliefs about Knowledge and Knowing.

[23] Lei H., Xu G., Shao C., Sang J. (2015). The relationship between teachers’ caring behavior and students' academic development: the mediating role of learning self-efficacy. Psychol. Dev. Educ..

[24] Cocoradă E. (2016). Achievement emotions and performance among university students. Bulletin of the Transilvania University of Braşov, Series VII: Social Sciences and Law.

The article "On the correlation among the students’ epistemic cognition, academic emotions, and academic achievement in higher education" was retracted in 2025. Reasons: plagiarized text; unreliable results or conclusions; concerns about the citations.

[25] Kim C., Hodges C.B. (2012). Effects of an emotion control treatment on academic emotions, motivation and achievement in an online mathematics course. Instr. Sci..

[26] Villavicencio F.T., Bernardo A.B. (2013). Positive academic emotions moderate the relationship between self-regulation and academic achievement. Br. J. Educ. Psychol..

[27] Lam U.F., Chen W.-W., Zhang J., Liang T. (2015). It feels good to learn where I belong: school belonging, academic emotions, and academic achievement in adolescents. Sch. Psychol. Int..

[28] Villavicencio F.T. (2011). Critical thinking, negative academic emotions, and achievement: a meditational analysis. The Asia-Pacific Education Researcher.

[29] Shen B., Wang Y., Yang Y., Yu X. (2023). Relationships between Chinese university EFL learners' academic emotions and self-regulated learning strategies: a structural equation model. Lang. Teach. Res..

[30] Greene J.A., Yu S.B. (2014). Modeling and measuring epistemic cognition: a qualitative re-investigation. Contemp. Educ. Psychol..

[31] Hofer B.K. (2004). Epistemological understanding as a metacognitive process: thinking aloud during online searching. Educ. Psychol..

[32] Hofer B.K. (2006). Beliefs about knowledge and knowing: integrating domain speciﬁcity and domain generality: a response to Muis, Bendixen, and Haerle (2006). Educ. Psychol. Rev..

[33] Hofer B.K., Bendixen L.D., Harris K.R., Graham S., Urdan T. (2012).

[34] Hofer B.K., Pintrich P.R. (1997). The development of epistemological theories: beliefs about knowledge and knowing and their relation to learning. Rev. Educ. Res..

[35] Hofer T., Pintrich P.R. (2002).

[36] Hofer B.K., Sinatra G.M. (2010). Epistemology, metacognition, and self- regulation: musings on an emerging ﬁeld. Metacognition & Learning.

[37] Sandoval W.A., Çam A. (2010). Elementary children's judgments of the epistemic status of sources of justiﬁcation. Sci. Educ..

[38] Buehl M.M., Alexander P.A. (2005). Motivation and performance differences in students' domain-speciﬁc epistemological belief proﬁles. Am. Educ. Res. J..

[39] Greene J.A., Muis K.R., Pieschl S. (2010). The role of epistemic beliefs in students' self-regulated learning with computer-based learning environ- ments: conceptual and methodological issues. Educ. Psychol..

[40] Perry W.G. (1968/1999).

[41] Lonka K., Ketonen E., Vermunt J.D. (2021). University students' epistemic profiles, conceptions of learning, and academic performance. High Educ..

[42] Tsai C.C., Liu S.Y. (2005). Developing a multi-dimensional instrument for assessing students' epistemological views toward science. Int. J. Sci. Educ..

The article "On the correlation among the students’ epistemic cognition, academic emotions, and academic achievement in higher education" was retracted in 2025. Reasons: plagiarized text; unreliable results or conclusions; concerns about the citations.

[43] Muis K.R. (2007). The role of epistemic beliefs in self-regulated learning. Educ. Psychol..

[44] Muis K.R. (2008). Epistemic profiles and self-regulated learning: examining relations in the context of mathematics problem solving. Contemp. Educ. Psychol..

[45] Arslantas H.A. (2016). Epistemological beliefs and academic achievement. Journal of Education and Training Studies.

[46] Greene J., Cartiff Brian M., Duk Rebekah F. (2018). A meta-analytic review of the relationship between epistemic cognition and academic achievement. J. Educ. Psychol..

[47] Muis K. (2007). The role of epistemic beliefs in self-regulated learning. Educ. Psychol..

[48] Muis K.R., Duffy M.C. (2013). Epistemic climate and epistemic change: instruction designed to change students' beliefs and learning strategies and improve achievement. J. Educ. Psychol..

[49] Schiefer J., Edelsbrunner P.A., Bernholt A. (2022). Epistemic beliefs in science—a systematic integration of evidence from multiple studies. Educ. Psychol. Rev..

[50] Guo X., Hao X., Deng W. (2022). The relationship between epistemological beliefs, reflective thinking, and science identity: a structural equation modeling analysis. International Journal of STEM Education.

[51] Madjar N., Weinstock M., Kaplan A. (2016). Epistemic beliefs and achievement goal orientations: relations between constructs versus personal profiles. J. Educ. Res..

[52] Lonka K., Ketonen E., Vermunt J.D. (2021). University students' epistemic profiles, conceptions of learning, and academic performance. High Educ..

[53] Otting H., Zwaal W., Tempelaar D., Gijselaers W. (2010). The structural relationship between students' epistemological beliefs and conceptions of teaching and learning. Stud. High Educ..

[54] Sadi Ö., Dağyar M. (2015). High school students' epistemological beliefs, conceptions of learning, and self-efficacy for learning biology: a study of their structural models. Eurasia J. Math. Sci. Technol. Educ..

